# Application Effect of External and Internal Elevation of Maxillary Sinus in Implant Restoration of Posterior Maxilla

This article has been retracted.

**DOI:** 10.1155/2022/7879633

**Published:** 2022-09-01

**Authors:** Xuan Deng, Rujie Shi, Jia Zhan, Fang Yang

**Affiliations:** ^1^The Second Affiliated Hospital, Department of Stomatology, Hengyang Medical School, University of South China, Hengyang, Hunan 421001, China; ^2^The Second Affiliated Hospital, Department of Neurosurgery, Hengyang Medical School, University of South China, Hengyang, Hunan 421001, China

## Abstract

**Objective:**

To explore and analyze the application effect of external and internal elevation of the maxillary sinus in implant restoration of the posterior maxilla.

**Methods:**

A total of 84 patients undergoing implant restoration of the posterior maxilla in the hospital were enrolled between January 2019 and March 2021. According to the random number table method, they were divided into the observation group (*n* = 42) and the control group (*n* = 42). The control group underwent external elevation of the maxillary sinus, while the observation group underwent internal elevation of the maxillary sinus. At 6 h, 12 h, and 24 h after surgery, the pain degree between the two groups was compared. All were followed up at 6 months after surgery. The osseointegration (bone resorption around implants, elevation height of maxillary sinus floor, average healing time) and soft tissues (bleeding index, plaque index, probing depth) in both groups were observed. The occurrence of postoperative complications was recorded.

**Results:**

At 6 h, 12 h, and 24 h after surgery, VAS scores in the observation group were significantly lower than those in the control group (*P* < 0.05). At 6 months after surgery, bone resorption and elevation height of the maxillary sinus floor in the observation group were significantly higher than those i.0.0n the control group, and the average healing time was significantly shorter than that in the control group (*P* < 0.05). The bleeding index, plaque index, and probing depth in the observation group were significantly lower than those in the control group (*P* < 0.05). There was no significant difference in the incidence of postoperative complications between the observation group and the control group (9.52% vs. 19.05%) (*P* > 0.05).

**Conclusion:**

The application effect of internal elevation of the maxillary sinus is good in implant restoration of the posterior maxilla, which can relieve pain and swelling and improve implant effect.

## 1. Introduction

Oral implant restoration has now become one of the important restoration methods for missing teeth. As an anatomical structure, the posterior maxillary area is complicated, and the restoration of this area is one of the most challenging surgical procedures in implant surgery [1]. Due to the particularity of the anatomical structure, the roots of the maxillary posterior teeth are closely connected to the maxillary sinus. In addition, some patients are often complicated by severe periodontitis or dental caries, resulting in the loss, loosening, or atrophy of the maxillary posterior teeth, which not only seriously affects the patients. The patient's quality of life and psychological state also increase the difficulty of implant placement in this dental area [2, 3]. In the past, the conventional implantation method was easy to penetrate until the mucosa of the maxillary sinus floor, resulting in the emergence of complications and affecting the surgical effect [4]. With the rapid development and progress of implant technology and medical technology, a maxillary sinus lift is widely known and used in clinics. This method includes maxillary sinus internal and external lifts. By increasing the bone height of the maxillary sinus alveolar, the purpose of implant restoration is achieved. This method can effectively improve the bone mass in the posterior maxillary area, reduce the occurrence of postoperative complications, and provide a guarantee for the corresponding function of dental implants. It has been widely used in clinical practice [5, 6]. But at present, there is no unified conclusion about the choice of its surgical method. Therefore, in this study, maxillary sinus lift was used in the implant restoration of maxillary posterior teeth in order to evaluate the effect of maxillary sinus internal and external lift in implant restoration of maxillary posterior teeth and to provide a theoretical basis for clinical selection of appropriate surgical methods.

## 2. Materials and Methods

### 2.1. General Information

A total of 84 patients who underwent implant restoration in the maxillary posterior region in our hospital from January 2019 to March 2021 were selected. The patients were divided into an observation group (*n* = 42) and a control group (*n* = 42) by the random number table method. The observation group included 23 males and 19 females, aged 26–49 years, mean age 37.73 ± 3.61 years old, body mass index of 18–22 kg/m^2^, and a mean age 20.13 ± 0.25 kg/m^2^. The control group consisted of 25 males and 17 females, aged 26–49 years, a mean age 37.41 ± 3.45 years old, body mass index 18–22 kg/m^2^, and a mean body mass index 20.22 ± 0.18 kg/m^2^. There was no significant difference in general data between the two groups (*P* > 0.05). This study was approved by the hospital ethics committee.

### 2.2. Inclusion Criteria

① All patients underwent routine CT examination before surgery and met the surgical indications for implant restoration in the maxillary posterior region [7]. ② The patients and their families understood and gave informed consent to this study. ③ The vertical distance from the maxillary sinus floor to the alveolar ridge top is ≥ 5 mm.

### 2.3. Exclusion Criteria

① Patients with adjacent periodontitis or apical lesions; ② patients with systemic diseases; ③ patients with confusion or mental illness; ④ patients with important organ disease; and ⑤ there are patients who cannot tolerate surgery.

### 2.4. Surgical Methods

Both groups of patients underwent routine CT examinations before the operation, and the implant position was determined in advance, the corresponding implant materials were prepared according to the CT examination results, and the patients were instructed to use mouthwash for oral cleaning. The patient was placed in a supine position and local anesthesia was administered.

The control group was treated with a maxillary sinus external lift. A trapezoidal incision was made on the top of the alveolar ridge at the defect of the patient's maxillary posterior teeth, and the mucoperiosteal flap was opened and peeled to expose the alveolar bone implantation area. Then, use a ball drill to prepare a hole, determine the scope of the opening, and cut open the anterior and lateral walls of the maxillary sinus to completely expose the maxillary sinus mucosa. Finally, implants and artificial bone powder are implanted, covered with an oral prosthetic membrane, and sutured layer by layer.

The observation group was treated with maxillary sinus internal lift. A horizontal incision was made on the alveolar crest and buccal side of the patient to open the mucoperiosteal flap to fully expose the lateral wall of the maxillary sinus. A ball drill was used to determine the scope and location of the window at about 5 cm above the implant site at the lower wall of the maxillary sinus., the window opening range is about 1.5 cm. Use a bone squeezer to lift the remaining bone plate together with the mucosa of the sinus floor, expand the implant area step by step, fill it in with the bone powder and implant, cover it with a prosthetic membrane, and finally close the surgical incision.

### 2.5. Observation Indicators

#### 2.5.1. Pain Level

At 6 h, 12 h, and 24 h after the operation, the visual analogue scale (VAS) [8] was used to evaluate the pain degree of the patients. The total score on the scale was 0–10 points. A higher score indicates more severe pain.

#### 2.5.2. Osseointegration Index

Six months after the operation, the Dutch oral panoramic X-ray machine was used to take pictures, and the bone resorption around the implants, the height of the maxillary sinus floor, and the average healing time of the implants were measured in the two groups of patients.

#### 2.5.3. Soft Tissue Conditions

One day before surgery and 6 months after surgery, a special periodontal probe was used to measure the distance from the gingival margin to the bottom of the gingival sulcus, which was the probing depth. The bleeding index and bacterial plaque index of the mesial, central, and distal parts of the lip and tongue were compared between the two groups, and the results were averaged. The bleeding index: 0 points: no bleeding; 1 point: punctate bleeding; 2 points: bleeding at the gingival margin. The plaque index: 0 points: no plaque; 1 point: the plaque can be detected by the probe; 2 points: Plaque was observed on the oral surface.

#### 2.5.4. Complications

Postoperative complications were recorded, including maxillary sinus mucosal perforation, local infection, implant loosening, pain, and swelling.

### 2.6. Statistical Processing

The SPSS 22.0 statistical software was used to process and analyze the data of this study, and the measurement data such as osseointegration index, soft tissue condition, VAS, and swelling degree score that satisfied normal distribution and homogeneous variance were expressed as ($\bar{x}$ ± *s*), The differences between the observation group and the control group without time points were compared using a two-sample independent *t*-test, and the differences between groups with time points were compared by repeated measures analysis of variance. Before and after surgery, the differences between the observation group and the control group were compared using paired *t*-test, the count data were expressed by *n* (%), and the chi-square test was used. *P* < 0.05 indicated that the difference was statistically significant.

## 3. Results

### 3.1. Comparison of Pain Scores between the Two Groups of Patients

The pain scores of VAS of the group treated with maxillary sinus internal lift at 6 h, 12 h, and 24 h after operation was significantly lower than that of the group treated with maxillary sinus external lift (*P* < 0.05), as shown in Figure 1.

### 3.2. Comparison of Osseointegration Index Levels between the Groups Treated with Maxillary Sinus External/Internal Lift of Patients

After the operation, the bone resorption volume and height of the patients in the group treated with maxillary sinus internal lift were significantly higher than those in the group treated with maxillary sinus external lift. The average healing time was significantly lower than that of the group treated with maxillary sinus external lift (*P* < 0.05), as shown in Figure 2.

### 3.3. Comparison of Soft Tissue Conditions between the Groups Patients Treated with Maxillary Sinus External/Internal Lift

Before surgery, there was no significant difference in the bleeding index, plaque index, and probing depth between the groups treated with maxillary sinus external/internal lift (*P* > 0.05). After the operation, the bleeding index, plaque index, and probing depth of the groups treated with maxillary sinus external/internal lift were decreased. The internal maxillary sinus lifting group was lower than the external maxillary sinus lifting group (*P* < 0.05) as shown in Figure 3.

### 3.4. Comparison of Postoperative Complications between the Groups Treated with Maxillary Sinus External/Internal Lift of Patients

The incidence of complications in the group treated with maxillary sinus internal lift was 9.52%, which was not significantly different from 19.05% in the group treated with maxillary sinus external lift (*P* > 0.05), as shown in Table 1.

## 4. Discussions

Due to the continuous gasification and expansion of the maxillary sinus, the distance between the top of the maxillary alveolar ridge and the bottom wall of the maxillary sinus is reduced, and the bone is more porous, resulting in a lower height of the remaining alveolar bone in the implant area, which is prone to atrophy, thus increasing the difficulty of dental implants [9, 10]. In recent years, the maxillary sinus lift has had a good clinical effect on the implant restoration of the maxillary posterior region. However, domestic and foreign scholars still have some controversy about the specific choice of maxillary sinus internal and external lift [11, 12]. By comparing the effects of internal and external maxillary sinus lifts on postoperative pain, swelling, osseointegration, and soft tissue, this study provides ideas for exploring the best surgical approach for a maxillary sinus lift.

Maxillary sinus lift surgery has the characteristics of large lifting space, easy control, a clear surgical field, and sufficient bone mass. However, because the natural roots of maxillary premolars and molars are often located in the maxillary sinus cavity, the maxillary sinus mucosa Surrounding the root of the tooth, walking irregularly, and the maxillary sinus itself is uneven, it is difficult to peel off the mucosa of the maxillary sinus intact under the influence of the adjacent roots in the near, far, and middle when the maxillary sinus floor lifting operation is performed after a single tooth or a missing spacer tooth [13, 14]. The maxillary sinus lift has the advantages of being a simple operation, less trauma, quick postoperative recovery, and no need for additional operations. The maxillary sinus floor is lifted to a certain height by a specific maxillary sinus internal lifting device, and the integrity of the maxillary sinus floor mucosa is ensured at the same time [15]. In this study, the VAS and swelling scores of the patients in the observation group were significantly lower than those in the control group (*P* < 0.05), suggesting that compared with the external maxillary sinus lift, the maxillary sinus lift has greater advantages in reducing postoperative pain and swelling. This may be due to the small surgical scope of maxillary sinus lift surgery only an incision is made at the top of the alveolar ridge, and the operation can be completed in a short time. It avoids the damage to the sinus floor bony mucosa by surgical instruments, reduces the damage to the surrounding tissues [16], and makes the postoperative pain and swelling of the patients less severe.

In this study, the amount of bone resorption and height of the patients in the observation group were significantly higher than those in the control group, and the average healing time was significantly lower than that in the control group (*P* < 0.05). Heal quickly. The reason for this may be that after the operation has pushed up the maxillary sinus mucosa, a space is formed here, where a large number of blood clots are gathered, and these blood clots provide a good condition and environment for the formation of new bone, which is conducive to stimulation. Osteogenic precursor cells in the periosteum form new bone. In addition, trauma caused by surgical trauma and heat generation in the preparation of the cave will lead to the appearance of an inflammatory response, which in turn induces the activation of osteoclasts and promotes bone resorption [17, 18]. At the same time, because the bone will cause bone resorption after being squeezed to a certain extent, the vertical height of the bone will be reduced, and when the implant is implanted for repair, the surrounding bone will be tighter and the bone resorption will be further increased [19]. In addition, the results of this study showed that the bleeding index, plaque index, and probing depth of the observation group were significantly lower than those of the control group (*P* < 0.05), suggesting that maxillary sinus lift was more helpful for the reconstruction of periodontal tissue in patients with implant restoration in the maxillary posterior region, reducing the damage to periodontal tissue. The bleeding index, plaque index, and probing depth were all sensitive indicators reflecting periodontitis. Lifting the maxillary sinus is beneficial to enhance the stability of the implant, avoid loosening and falling off, and thus reduce the probability of infection, which is of great significance to protect the health of periodontal tissue, reduce the formation of periodontal plaque, and reduce the appearance of swelling and bleeding. In addition, this study showed no difference in the incidence of complications between the two groups. However, both groups experienced maxillary sinus mucosal perforation, pain, and swelling after surgery, all of which were common complications of maxillary sinus elevation. Among them, patients with perforation of maxillary sinus mucosa had relatively small perforations, no local infection symptoms, and self-cured through the self-repair function of the human body without causing serious adverse effects. The pain and swelling were also improved after the proper intervention. However, this suggests that attention should also be paid to the possible complications in the dental implant-supported restoration of the maxillary posterior region in the clinic, and we should be vigilant about the effects of various complications on the prognosis.

In conclusion, compared with the maxillary sinus lift, the maxillary sinus lift has a better application effect in the implant restoration of the maxillary posterior region, which can reduce the damage to the periodontal tissue and reduce the postoperative pain and swelling. It has a positive significance for promoting bone resorption and increasing the height of the maxillary sinus floor. At the same time, it has high safety and is worthy of widespread clinical application. The disadvantage of this study is that the included sample size is too small and the results have selection bias. The clinical sample size should be expanded for more in-depth research to confirm.

## Figures and Tables

**Figure 1:** Comparison of pain scores between the groups treated with maxillary sinus external/internal lift. Note. Compared with the group treated with maxillary sinus external lift, ^*∗*^*P* < 0.05.

**Figure 2:** Comparison of bone binding indexes between the groups treated with maxillary sinus external/internal lift. Note. Compared with the group treated with maxillary sinus external lift, ^*∗*^*P* < 0.05.

**Figure 3:** Comparison of soft tissue between the groups treated with maxillary sinus external/internal lift. Note: Compared with preoperative, ^*∗*^*P* < 0.05.

**Table 1:** Comparison of postoperative complications between the groups treated with maxillary sinus external/internal lift (*n* = 42, %).

Groups	Maxillary sinus mucosa perforation	Local infection	Implant loosening	Pain	Swell	Normal tissue complication probability
Observation group	2 (4.76)	0 (0.00)	0 (0.00)	1 (2.38)	1 (2.38)	4 (9.52)
Control group	1 (2.38)	2 (4.76)	1 (2.38)	2 (4.76)	2 (4.76)	8 (19.05)
*χ* ^*2*^	—	—	—	—		0.7117
*P*	—	—	—	—		0.397

## Data Availability

The data can be obtained from the author upon reasonable request.
